The article "Psychobiobehavioral Model for Preterm Birth in Pregnant Women in Low- and Middle-Income Countries" was published in 2015. Journal: Biomed Res Int.

# Psychobiobehavioral Model for Preterm Birth in Pregnant Women in Low- and Middle-Income Countries

**DOI:** 10.1155/2015/450309

**Published:** 2015-08-27

**Authors:** Shahirose S. Premji, Ilona S. Yim, Aliyah Dosani (Mawji), Zeenatkhanu Kanji, Salima Sulaiman, Joseph W. Musana, Pauline Samia, Kiran Shaikh, Nicole Letourneau, MiGHT Group

**Affiliations:** ^1^Faculty of Nursing, University of Calgary, 2500 University Drive NW, Calgary, AB, Canada T2N 1N4; ^2^Department of Community Health Sciences, Faculty of Medicine, University of Calgary, TRW Building, 3rd Floor, 3280 Hospital Drive NW, Calgary, AB, Canada T2N 4Z6; ^3^Alberta Children's Hospital Research Institute for Child and Maternal Health, Heritage Medical Research Building, 3330 Hospital Drive NW, Calgary, AB, Canada T2N 4N1; ^4^O'Brien Institute for Public Health, University of Calgary, 3280 Hospital Dr NW, Calgary, AB, Canada T2N 4Z6; ^5^Department of Psychology and Social Behavior, University of California, Irvine, 4562 Social and Behavioral Sciences Gateway, Irvine, CA 92697-7085, USA; ^6^School of Nursing and Midwifery, Mount Royal University, 4825 Mount Royal Gate SW, Calgary, AB, Canada T3E 6K6; ^7^School of Nursing and Midwifery, Aga Khan University-East Africa, Opposite Aga Khan Primary School Plot (9/11), Colonel Muammar Gaddafi Road, P.O. Box 8842, Kampala, Uganda; ^8^School of Nursing and Midwifery, Aga Khan University-Karachi, Stadium Road, P.O. Box 3500, Karachi 74800, Pakistan; ^9^Department of Obstetrics & Gynecology, Faculty of Health Sciences, Aga Khan University-Nairobi, 3rd Parklands Avenue off Limuru Road, P.O. Box 30270, Nairobi 00100, Kenya; ^10^Department of Pediatrics, Aga Khan University-Nairobi, 2nd Parklands Avenue, East Tower Block, Room 505, Nairobi 00100, Kenya

## Abstract

Preterm birth (PTB) is a final common outcome resulting from many interrelated etiological pathways; of particular interest is antenatal psychosocial distress (i.e., stress, anxiety, and depression). In LMI countries, both exposure to severe life stressors and rate of PTB are on average greater when compared with high-income countries. In LMI countries women are exposed to some of the most extreme psychosocial stress worldwide (e.g., absolute poverty, limited social resources). High prevalence of antenatal stress and depression have been observed in some studies from LMI countries. We propose a psychosocial, biological, and behavioral model for investigating the complex multisystem interactions in stress responses leading to PTB and explain the basis of this approach. We discuss ethical considerations for a psychosocial, biological, and behavioral screening tool to predict PTB from a LMI country perspective.

## 1. Introduction

Preterm birth (PTB) is a global health concern with a worldwide prevalence rate exceeding 10%. PTB is associated with a high rate of death in the first year of life accounting for 80% of the world's 1.1 million deaths of children, as well as 50% of pediatric neurodevelopment problems [1–4]. Twelve of the 15 countries that contribute more than 60% to the global burden of PTB are low- and middle-income (LMI) countries [1]. Pakistan, Kenya, and the United Republic of Tanzania (hereafter Tanzania), for instance, have a PTB rate of 15.8, 12.3, and 11.4 per 100 live births, respectively [5]. We use these countries as exemplars when presenting perspectives on antenatal psychosocial distress (i.e., emotional suffering presenting as depression and anxiety during pregnancy) and pathways to PTB. Despite the higher incidence of both PTB and psychosocial distress in many LMI countries, empirical work on psychosocial predictors of PTB has been predominantly conducted in high-income countries [6, 7]. While this body of research is very valuable, findings are not necessarily applicable to LMI countries.

How do LMI countries differ from high-income countries in ways that may influence the link between stress and PTB? Most obviously, family resources are generally limited as a result of poverty, which restrict women's ability to seek care during and following birth [8]. Women in LMI countries, for instance, Pakistan, are exposed to greater poverty with 17% of the population living below the poverty line (2007/8 statistics) [9]. Existing resources must be conserved for basic care for the child and often simply for survival. Poor quality of care in facilities which are not well resourced and poor attitude of staff [8] may amplify women's fears about pregnancy being risky both for them and their infants. Moreover, every day approximately 800 women die as consequence of pregnancy- or childbirth-related problems; almost all of these deaths are situated in LMI countries [10]. Similarly, almost all neonatal deaths occur in LMI countries and predominantly in the neonatal period, that is, within the first four weeks following birth. During the postpartum period, limited care and resources are available to women and their babies.

Second, exposure to severe life stressors (e.g., absolute poverty, limited social resources) is on average greater in LMI countries, compared to high-income countries. High prevalence of antenatal stress and depression have been observed in some studies from LMI countries (e.g., 40.9% in a secondary hospital based sample [11] and 25% in a community-based sample [12]). These rates are comparable to subpopulations of low socioeconomic North American and European women (e.g., 23–47%) [13, 14]. The exposure to more and more intense stressors among women in LMI countries is likely not without consequence. Maternal psychosocial distress (i.e., pregnancy-related anxiety, state anxiety, depression, or perceived stress) during pregnancy has been linked to PTB [14–16]. Moreover, both PTB and psychosocial distress are associated with offspring's negative lifelong developmental and intergenerational trajectories and may have a disproportionate toll in LMI countries.

A final difference is that pregnant women in LMI countries are bound by different social norms and cultural ties. Women in LMI countries experience inequities in access to education (43% literacy rate for males compared to 28% for females) [17] and economic opportunities. In many cases, sociocultural norms in LMI countries may limit women's ability to act autonomously or have a voice in care decision [18]. Pregnant women worry about sex of their unborn infant as male preference is common. For instance, in Pakistan, a women's status within the family may be linked to birth of a son [11, 17–19]. The importance attached to a male child [20] limits their opportunity to be involved in decision-making and creates dynamic social relations within the family in relation to both their own care and their infant [18].

In sum, while PTB is particularly prevalent in many LMI countries, LMI countries lag behind in explicating the contribution of psychosocial distress to PTB and where limited resources are available to translate empirically derived knowledge into prevention. We propose a model including psychosocial, biological, and behavioral dimensions to investigate the complex multisystem interactions linking stress with PTB with a particular emphasis on LMI countries. Conceptualizing the stress-PTB link in LMI countries will not only allow us to gain insight into psychosocial predictors of PTB in LMI countries but also provide unique opportunities to improve our understanding of the etiology of PTB. We discuss the potential benefits and limitations of developing a population-based psychosocial, biological, and behavioral screening tool to predict PTB from a LMI country perspective, given existing resources.

## 2. Materials and Methods

We searched peer-reviewed electronic databases (MEDLINE, Embase, Global Health, and Cumulative Index to Nursing and Allied Health Literature), grey literature, and reference list of relevant articles, as well as solicited articles from an existing peer network in Pakistan, Kenya, and Tanzania. The details of the search and selection strategy, quality assessment and data extraction, and consultation exercise are described in detail elsewhere [21]. To explicate the potential benefits and limitations of developing a population-based psychosocial, biological, and behavioral screening to predict PTB from a LMI country perspective, a new search strategy was undertaken. Key terms such as prediction, mass screening, and serum screening were combined with pregnancy outcome; stress, psychological; and preterm birth. No limits were applied with regard to country of origin of studies or language. The synthesis of the literature shared below draws from the realist approach in recognition that systematic reviews often exclude important observations from studies deemed less rigorous that may illuminate “mechanisms” [22–24] or pathways to PTB. The realist approach relies on the expertise of those undertaking the review to build an explanatory theory (i.e., how and why) of the observed impacts and provide insight and identify gaps and mechanisms that need to be explored [22–24]. Our Maternal Infant Global Health Team (Global Collaborators in Research) (MiGHT) includes clinicians (e.g., nurse, midwife, obstetrician and gynecologist, psychologist, and laboratory specialist), researchers, and policy decision makers who have critically evaluated the literature. The breadth in the synthesis is the result of (a) situating our observations of behavioral practices such as pica or the deliberate consumption of soil and (b) revisiting the literature to deconstruct the nature of stress (e.g., chronic, acute) and (c) offering potential explanations for the varied findings in studies examining the relationship between psychosocial distress and PTB.

## 3. Results and Discussion

Our initial conceptual framework [21] on the relationship between psychosocial distress and PTB continues to evolve.  Figure 1 reflects our refined understanding of environment stressors pregnant women in LMI countries are exposed to and their response to this environment. Our new model specifically considers (a) individual differences in stress reactivity and accounts for the fact that not all women who experience psychosocial stressors will have an adverse pregnancy outcome, (b) biological response patterns expressed as a cumulative physiologic burden (i.e., allostatic load), (c) behavioral response patterns to stress, and (d) interactive feedback effects. The model exemplifies the importance of early identification of psychosocial stressors and maladaptive biological and behavioral responses given the interplay of multiple systems in the pathways to PTB.

### 3.1. Conceptual Framework

Below we discuss each concept of the model followed by implications of developing a population-based screening tool based on the psychosocial, biological, and behavioral model. We conclude by offering highlights of the importance and relevance of this work.

#### 3.1.1. Stress-Related Physiological Responses and Biological Mediators of PTB: Racial Differences

Independent risk factors for PTB account for less than half of the racial disparity in risk of PTB, particularly between black and white women in United States of America, the former having a higher risk of delivering very preterm [25]. Medical conditions of pregnancy, for example, gestational hypertension and preeclampsia, have also been shown to differ by ethnic background after adjusting for socioeconomic and other risk factors within social context (e.g., education level, lifestyle-related factors) [25–29].

In the nonpregnant state, biological responses to stress (e.g., physical exercise), specifically the release of cortisol and adrenocorticotropic hormone, differed between African American and Caucasian women, such that Caucasian women showed higher levels of adrenocorticotropic hormone without associated increases in cortisol [30]. Ethnic differences in hypothalamic-pituitary-adrenal (HPA) axis functioning have also been found in pregnant women [31–33]. During pregnancy, biomarkers (e.g., cortisol, adrenocorticotropic hormone, corticotropin-releasing hormone, nonfasting cholesterol, and triglyceride levels) and trajectories of biomarkers (e.g., corticotropin-releasing hormone) of the HPA system have been reported to differ by ethnicity after accounting for risk factors (e.g., socioeconomic and behavior) [31–35]. An earlier systematic review reported an association between race/ethnicity and C-reactive protein level after adjusting for confounding (e.g., age, sex) and mediating (e.g., obesity, smoking) variables [36]. South Asian cohorts had higher levels of C-reactive protein than Caucasian women (i.e., white) [36]. The magnitude of changes in stress-related physiological measures across pregnancy and biological mediators of PTB also differ depending on race/ethnicity [37–39]. For example, African American women have lower levels of cortisol during early gestation (i.e., 18–20 weeks of gestation) than non-Hispanic white women and the lowest increase in corticotropin-releasing hormone over the course of pregnancy (24–26 and 30–32 weeks of gestation) [31]. Moreover, a “Hispanic paradox” has been observed whereby better pregnancy outcomes have been reported among Hispanic women despite severe preeclampsia and adverse sociodemographic profiles [40]. Although the underlying pathways remain unknown, it has been proposed that biological systems (e.g., cardiovascular) of ethnic groups may adapt differently given environmental differences [27, 41, 42].

#### 3.1.2. Acute Stress and Chronic Stress

Stress is defined “as an imbalance between demands placed on us (from our environment) and our ability to manage them” [43, page 121] which manifests as psychosocial distress. Psychosocial distress is multifaceted and encompasses emotional states that result from acute stress (e.g., a heated argument with spouse, divorce, and loss through death), emotional states that characterize the individual (e.g., anxiety, depression), and chronic stressors experienced as a consequence of social, cultural, and environmental phenomena [44, 45]. Acute stress is deemed to be short term, though no operational definition is provided for “short,” and allows the body to regain homeostasis [45, 46]. Pregnancy itself may be viewed as an acute stressor in a sense that it may elicit fears of maternal and neonatal mortality and morbidity particularly surrounding delivery and the forthcoming responsibility of providing for a child, a concept that has been referred to as pregnancy-related anxiety [47]. In contrast, chronic stressors are those where the threat or demand persists over time; that is, they are long-lived and resolution may or may not be achieved [44, 46]. Chronic stress may partly reflect external events that are enduring sources of stress in day-to-day life such as neighborhood crime, poverty, homelessness or household strain, and racial composition [44]. It is beyond the scope of this paper to synthesize the literature on each dimension of psychosocial distress; however, we present below a brief overview.

Psychosocial distress is associated with pregnancy outcomes, controlling for other risk factors including, for example, health behaviors, medical, and sociodemographic factors [45, 48]. The magnitude of the effect, however, seems to vary by location of study (high- versus low-income) [16], socioeconomic status (United States) [16], ethnic and immigrant populations, and periods of gestation [37]. Moreover, in studies from high-income countries, dimensions of psychosocial distress were noted to exert differential influences on PTB. Pregnancy-related anxiety consistently predicts PTB and this association is evident in diverse income and ethnic groups [15]. North American and European studies examining the relationship between depression and PTB have also shown inconsistent findings, with a minority of the studies finding (e.g., [49–51]) a statistically significant association with a small effect size [15]. Though many North American and European studies have shown an association between state anxiety or emotional response due to situational circumstances (e.g., fear or danger due to catastrophic events) and PTB (e.g., [15, 50, 52]), findings have been mixed, with studies demonstrating no association (e.g., [53, 54]) and associations in subgroups of samples or in combination with other measures [15]. Similarly, a person's perception of ongoing and enduring sources of stress in their day-to-day life has shown mixed results with large studies reporting an association (e.g., [55]) as well as no association (e.g., [14]) with PTB.

We proposed that the impact of stress on PTB involves intersects between acute and chronic stress (i.e., multidimensional nature of stress) and biological (i.e., biomarkers) and behavioral responses that establish differential pathways to PTB [25, 45]. For instance, childhood adversity increases vulnerability to adverse psychological (e.g., depression), physical (e.g., diabetes), and pregnancy (e.g., PTB) health outcomes [56–58]. Consequently, our model draws from the adverse childhood experiences-international questionnaire (ACE-IQ) which is intended to measure chronic stress in early life in individuals irrespective of country of domicile [59]. The individual (e.g., sexual and emotional abuse and neglect by parents or caregivers), social relationship (e.g., family dysfunction), sociocultural (e.g., race/ethnicity, socioeconomic status), and community level (e.g., witnessing community violence) items of the ACE-IQ [59], however, have not been validated. Examples of types of stressors within each level contributing to chronic stress are detailed in Figure 2 and many (e.g., education, socioeconomic measure, and domestic violence) have individually been associated with poor pregnancy outcome [47, 60–65]. Given “wear and tear” on the brain and body from these cumulative stressors (i.e., chronic stress), biological responses in multiple systems (e.g., HPA axis, cardiac, immune, and metabolic) may be compromised or fail outright. Increase in the individual's allostatic load as a consequence of dysregulation of these interrelated systems may ultimately result in pathophysiological effects, including PTB [66–68]. Our conceptual model also emphasizes the multiplicative nature of these responses to explain the pathogenesis of stress-related medical conditions during pregnancy which leads to induced PTB. Aspects of the HPA axis and sympathetic, immune, and cardiovascular systems also promote behavior changes in the effort to restore allostasis [46, 67]. Below we explain assertions and propose hypotheses for consideration for future research.

*Chronic Stress Influences Response to Acute Stress and Biomarkers Vary by Type of Stress*. Kramer et al. [25], drawing from studies in psychiatry (e.g., [69, 70]) and international migration and birth outcomes (e.g., [71]), have proposed that early life experiences can have long-term effects on the HPA axis, such as altering cortisol responses to acute stressors and baseline cortisol levels. For example, Finnish children separated from their fathers serving in World War II evidenced higher salivary cortisol and plasma adrenocorticotropic hormone in responses to a standardized psychosocial stress test more than 60 years after the separation. Baseline cortisol was significantly higher among separated women than nonseparated women who did not differ significantly in characteristics from separated women [70]. Early life experiences can also influence reactivity and biological responses to new stressful stimuli (e.g., pregnancy itself) [25, 69, 72]. For example, a systematic review of 24 studies (30 million singleton births) examining international migration and adverse birth outcomes reported lower risk of PTB among black immigrants when compared to black women born in the United States. In contrast, this level of protection was not conferred to Asian women who were at higher risk of PTB when compared to native-born population regardless of continent (e.g., United States and Europe) [71].

In epidemiological and clinical research, C-reactive protein is an important marker for a range of disease outcomes (e.g., cardiovascular, type 2 diabetes) [73]. Studies [74–76] indicate that CRP measured during early pregnancy is a useful predictor of PTB, particularly at specific cut-offs (e.g., greater than 4 mg/L [74]). The nature of stress (acute versus chronic) influences C-reactive protein levels [25, 72]. Chronic stress suppresses immune function or alters immune responses while acute stress stimulates immune function [25]. Inflammatory biomarkers have been shown to mediate the relationship between psychosocial stress (acute and chronic) and PTB [77, 78]. Interactions between acute and chronic stress influence C-reactive protein levels (and HPA axis functioning) suggesting that the impact of acute stress (e.g., pregnancy-related anxiety) can be amplified in the presence of chronic stress [72, 79]. Acute stress in combination with chronic stress may increase the strength of association with PTB [79]. C-reactive protein may improve risk stratification of PTB when combined with other biomarkers of PTB [80].

#### 3.1.3. Stress Reactivity

Many studies show an association between stressors experienced during pregnancy and PTB, but it is also clear that not all women exposed to stress during pregnancy will proceed to deliver preterm. This may be the case because of differences in how women* respond* to stressful situations they encounter. Support for this view comes from the broader literature on stress and disease suggesting that heightened psychobiological stress reactivity may explain, at least in part, why some but not all individuals exposed to stress will develop disease [81–83]. Below we highlight this literature. A broader review of the implications of individual differences in physiological stress reactivity for maternal and fetal birth outcomes is provided elsewhere [45].

There are only a handful of studies to date that have empirically tested the link between stress reactivity and birth outcomes, but they converge to suggest that more pronounced heart rate and blood pressure responses to laboratory stressors are associated with poorer birth outcomes. In the earliest of these studies, McCubbin et al. [84] assessed 39 primigravidae, predominantly white and black US women's heart rate and blood pressure responses to a computer-based arithmetic stressor protocol at approximately 35 weeks of gestational age. Findings suggest that women who proceed to deliver preterm had significantly higher diastolic stress responses than women with term infants. Moreover, each 1 mm Hg increase in diastolic reactivity was associated with a 0.31 weeks' decrease in gestational length. Similarly, de León et al. [85] reported a 0.07 weeks' decrease in gestational length with each 1 mm Hg increase in mean blood pressure in 70 pregnant Argentinian women exposed to the cold pressor test. That study also reported the absence of a link between baseline blood pressure and gestational length, highlighting the need to obtain stress reactivity measures. A third, larger study exposed 75 black and 238 white pregnant women to a mental arithmetic and Stroop color-word task [86]. For black women only, an association between a 1 mm Hg increase in diastolic reactivity and a decrease of 0.17 weeks of gestational length was observed. This finding indicates that stress reactivity may be an important variable to consider in studies aiming to explain the typically higher rate of PTB among black women [25, 87]. A final study is unique in that it assessed stress reactivity not during pregnancy but before pregnancy onset. Harville et al., [56] in a large, longitudinal study, tested the association between blood pressure responses to a video game, star tracing, and cold pressor test and preterm birth incidence in a first pregnancy occurring within 18 years after the stress exposure. Women with higher mean arterial pressure reactivity had higher PTB risk, suggesting that it is not only pregnancy-related increased blood pressure reactivity [84–86] that is associated with PTB but an underlying more general stress reactivity trait that maybe associated with poor birth outcomes.

*Allostatic Load and Its Biomarkers Predict PTB*. Psychosocial distress activates physiological responses in the HPA axis and sympathetic, immune, and cardiovascular systems in the effort to restore allostasis (i.e., physiological stability by altering the internal milieu) [46, 67]. In this context, biomarkers that detect physiological compromise might be useful as predictors of psychosocial distress and its negative consequences. Systematics reviews, however, have concluded that no single biomarker consistently predicts PTB and findings remain inconsistent [88, 89]. Allostatic load links psychosocial distress and its physiological responses over time, given “wear and tear” to multisystem dysregulation, which promotes a cascade of events ultimately impacting pregnancy outcome (i.e., PTB) [66–68, 90, 91]. Consequently, composite measures of biomarkers versus individual biomarkers may be a stronger predictor of negative consequences of psychosocial distress [92–94]. Despite the popularity of allostatic load as a research concept of stress in the general population and different allostatic load algorithmic computations available in the literature [94–96], only one small North American study was identified in the pregnancy-related field. In this study, secondary analysis of previously collected biomarkers showed an association between allostatic load at 26–28 weeks of gestation and gestational age [97]. An allostatic load index, in which a *z*-score of each biomarker was included, was inversely related to gestational age [97]. Interrelated physiological (i.e., biochemical) response patterns expressed as a cumulative physiologic burden, that is, allostatic load, may predict PTB and mitigate or exacerbate negative consequences of pregnancy-related anxiety. We moreover propose that biomarkers selected in future prospective studies should (a) represent patterns of events leading to allostatic load, (b) be empirically linked to psychosocial distress, and (c) be implicated in the pathophysiological processes linking perinatal distress to PTB. In the context of LMI countries, biomarkers should be easily obtained (e.g., serum versus cervicovaginal or amniotic fluid) and are amenable to point-of-care testing and of clinical utility to varied cadre of health care providers (e.g., midwives, skilled birth attendants) to facilitate immediate decision-making.

*Allostatic Load Explains Medically Induced PTB*. Pregnancy-induced hypertension and gestational diabetes are not only common during pregnancy but also the leading global causes of maternal and infant mortality and establish health trajectories over the course of life and across generations [98, 99]. In LMI countries, the incidence of preeclampsia is 2.8% of live births, notably seven times higher than in high-income countries [100, 101]. Although the incidence of gestational diabetes remains unknown, the high prevalence and growing incidence of diabetes in African populations, projected to 18.6 million by 2030, suggest that pregnant African women are at higher risk of gestational diabetes [102, 103]. Both preeclampsia and gestational diabetes form part of the indications for early delivery, hence PTB, and represent dysregulation in physiological processes which may in part be explained by allostatic load [104, 105].

Mood and anxiety disorders in women of childbearing age, either preconception or before 20 weeks of gestational age, increased risk of preeclampsia after controlling for variables such as age, race/ethnicity, and prepregnancy body mass index [106]. Moreover, allostatic load index ascertained using biomarkers—systolic blood pressure, diastolic blood pressure, pulse pressure, prepregnancy body mass index, total cholesterol, high-density lipoprotein, nonfasting triglyceride, C-reactive protein, and interleukin-6—measured prior to 15 weeks of gestational age was associated with preeclampsia [105]. During pregnancy, physiological regulatory set points (e.g., levels of insulin, cortisol, glucose, and leptin) continually change to accommodate the demands of the fetal-placental-maternal unit. Dysregulation of this complex metabolic system as a result of chronic insult such as stress and anxiety can explain the genesis of gestational diabetes and eventual type 2 diabetes [104]. Women who are metabolically challenged in early pregnancy (12 weeks), as indicated by increased levels of glycated hemoglobin [107], may present with hyperinsulinism, insulin insensitivity, and slighter high blood pressure prior to developing pregnancy-induced hypertension [99]. Increased glycated hemoglobin has been associated with adverse pregnancy outcomes (e.g., hypertension, miscarriage, and perinatal mortality) [107]. A relationship has been demonstrated between high diastolic blood pressure responses to stress during pregnancy and decreased gestational age [84–86]. It appears that women at risk of psychosocial distress who are also likely to develop pregnancy-induced medical conditions suggested the same etiologic entities with common terminal pathways for medically indicated and spontaneous preterm labor without premature rupture of chorioamniotic membranes [46, 93, 108–110]. Consequently, both subtypes should be examined in studies elucidating psychosocial distress and their biological pathways to PTB.

*Psychosocial Distress and Biomarkers Should Be Measured Repeatedly*. Pregnant women demonstrate a decrease in perceptions of psychosocial distress and dampening of biological stress responses in the late second trimester which is thought to protect the women and fetus [111]. Pregnant women who fail to demonstrate these changes may be at greater risk of PTB [37, 112]. Studies (e.g., [32, 111]) found that although point measures reported no association, changes in state anxiety [111], magnitude of change in perceived stress scale scores [32], and simply an increase in perceived stress [111] predicted either length of gestation [32] or PTB [111]. Glynn et al. [111] found that, in a regression model, pregnant women with increases in perceived stress were more likely to have a PTB than women with increase in state anxiety, although both are unique predictors of PTB. Similarly, decrease in triglyceride level with increasing gestational age has been implicated in PTB [113]. A slower increase in triglyceride level was noted in women who delivered prior to 34 weeks of gestation [114]. Point measures may therefore be of limited use to our understanding of the relationship between psychosocial distress, biomarkers, and PTB as psychosocial distress and biomarker measures are influenced by timing of pregnancy [37, 48, 111].

*Health Behaviors Compensate for Allostatic Load*. Health behaviors may be a means of compensating for allostatic load resulting from psychosocial distress to ensure stability, that is, allostasis [46, 115]. Psychosocial health during pregnancy has been linked to pica, the practice of eating nonnutritive substances (e.g., soil, raw starch, ice, and charcoal) for greater than 1 month [116, 117]. In many East African regions, women eat “odowa” (soft stones), “pemba” (white clay), or “udongo” (red clay), which can be purchased at local shops or markets [118, 119]. Approximately 45% of pregnant women attending antenatal clinics in Geita district, Mwanza, Tanzania, or health centre in western Kenya were practicing pica (i.e., eating soil) [118, 119]. However, rates as high as 63.7% have been reported in health facilities in Dar es Salaam, Tanzania [120].

While the prevalence of pica is high among women living in low- and middle-income countries [118–120], there is little information regarding the effects of this pregnancy-related behavior on PTB. Kawai and colleagues [121] found no association between geophagy and PTB as well as other pregnancy outcomes (e.g., small for gestational age and low birth weight). Studies, conducted in Argentina [122] and in Texas [123] and New York City in the United States [124], examining pica practices in relation to iron status and neonatal outcomes [122], maternal hemoglobin at delivery and pregnancy outcomes [123], and elevated lead levels [124] showed no statistical significant differences in rates of PTB [122, 123] or higher rates of preterm birth in pica practicing pregnant women [124].

Psychosocial distress has also been linked to addictive behaviors such as alcohol consumption. In Kenya, alcohol abuse is a mounting concern and is reported to be more prevalent than smoking [125, 126]. Factors contributing to increase in alcohol include socioeconomic challenges [125, 126] against a backdrop of changes in sociocultural norms [126]. Of particular concern are those who report drinking excessively, including women of child bearing age [125]. The Kenya Demographic and Health Survey indicates that unplanned pregnancies (defined as mistimed or unwanted) are common among unmarried Kenyan women 15–19 years of age and married Kenyan women [127, 128]. Pregnancy recognition may not occur for 5 weeks, during which time alcohol use may be high and lead to lifelong adverse consequences for the fetus (e.g., growth deficit, dysmorphology, and executive functioning, neuromotor, emotional, and speech/language difficulties) [129]. Over and above the direct effects of alcohol on the fetus, heavy maternal consumption of alcohol during pregnancy (i.e., dose response) has been associated with PTB [130–132]. The studies examining associations between alcohol consumption and PTB have been based in high-income countries (e.g., Australia, United States, Canada, and Spain).

### 3.2. Screening Programs

In LMI countries, the antenatal period provides the greatest opportunity for contact with women of reproductive age as more women seek care during pregnancy than preconception and in the postpartum period. Preconception care, that is, care initiated one year prior to the initiation of unprotected sexual intercourse, is routinely not offered or not accessible [133]. Although only 28% of pregnant women in Pakistan, and 47% in Kenya, receive antenatal care at least four times during pregnancy as recommended by the World Health Organization [134], the majority make at least one visit to an antenatal clinic: 61% in Pakistan and 92% in Kenya [135]. An integrated screening tool that considers psychosocial, biological, and behavioral measures to predict PTB has the potential to reduce psychosocial distress by implementing relatively low-cost psychological interventions early in pregnancy and improve pregnancy and health outcomes of mother and fetus/infant across the life span. Pakistan, like many other LMI countries, has minimal mental health resources; the services that are available are disorganized with respect to the catchment areas they serve [136]. In the absence of mechanisms to refer women to specialized health services (i.e., mental health and high risk pregnancies), costs would outweigh the benefits of screening [137]. Consequently, the psychosocial-biobehavioral screening tool will need to be administered by health care providers trained in perinatal mental health, be user friendly, and be implemented within a model of care that permits triaging high risk women, monitoring, or referring high risk women to appropriate mental health services [138].

The LMI country context requires special consideration in anticipating potential ethical challenges regarding psychosocial interventions. The sociocultural milieu influences women's care seeking behavior [18]; thus, ethical obligations to respect patient autonomy and to act with beneficence (i.e., do no harm) when promoting women's mental health [137] are much more complex given the dynamic nature of the decision-making. Designing and evaluating the effectiveness of a screening program must involve a community-based participatory approach in which stakeholders (i.e., pregnant women, families, and community leaders mutually) consider the social determinants of health to cocreate screening programs that will be taken up by the community [139, 140]. The approach espouses to the Public Health Code of Ethics which will advocate for and empower pregnant women with limited decision-making capacity to access health care services that are responsive to their needs [140].

Ethical approaches to managing clinical dilemmas with screening for psychosocial distress and risk of PTB must consider interrelationship between maternal mental health and fetal well-being, that is, relational ethics [137]. Allostatic load may indirectly influence maternal and infant health by impacting behavior systems thereby hindering mother-infant interactions [68, 90, 141]. These altered interactions in the long-term lead to delays in the infant's physical (i.e., growth, illness like diarrhea), emotional, cognitive, language, and social functioning [142–146] which can influence well-being of the mother, father, and family. Consequently, health care providers have an obligation to care for the mother (i.e., beneficence) as well as the fetus/infant (i.e., nonmaleficence or do no harm) [137].

## 4. Conclusion

The psychosocial, biological, and behavioral model proposed in this paper is unique as it considers each individual's unique life course that would influence stress perspective, biological responses, and coping strategies. Moreover, intervention strategies may be tailored to the risk profile identified thereby conserving and effectively utilizing limited resources in LMI countries. The model also stresses the importance of screening at multiple time points along the continuum of pregnancy as physiological processes of pregnancy alter stress responses (psychosocial and biological). The more blunted responses as pregnancy progresses protect the fetus and mother from adverse health consequences [37, 48, 111]. Key issues currently include identifying evidence-informed integrated psychosocial distress measures, biomarkers of allostatic load, and health behaviors; critical time periods for screening; and assessment and referral practices in poor resourced settings such as LMI countries.

## Figures and Tables

**Figure 1:** Psychosocial, biological, and behavioral model.

**Figure 2:** Chronic stress, types of stressors.
